RETRACTED

# A Retrospective Study on the Efficacy of Two Different Rehabilitation Interventions on KOA: Shock Wave Therapy vs. Electroacupuncture Therapy

**DOI:** 10.1155/2021/2099653

**Published:** 2021-11-29

**Authors:** Yuhui Zhao, Xuebing Wang, Dianquan Zhang

**Affiliations:** Rehabilitation Department, Shenzhen Longhua District Central Hospital, Shenzhen Guangdong Province, China 518110

## Abstract

**Objective:**

In this paper, we retrospectively reviewed the difference in clinical effectiveness of shock wave therapy and electroacupuncture therapy on knee osteoarthritis.

**Methods:**

A total of 128 treatment cases of knee osteoarthritis patients were extracted from the medical record system of Shenzhen Longhua District Central Hospital during the period from January 1, 2018, to January 30, 2020. The cases were divided into three groups for different treatments: shock wave group (*n* = 54), electroacupuncture group (*n* = 41), and control group (*n* = 33). The shock wave group was given shock wave therapy combined basis clinical treatment; meanwhile, the electroacupuncture group was given electroacupuncture on the basis of actual clinical treatment. The control group was given conventional topical nonsteroidal anti-inflammatory drugs (Voltaren). Osteoarthritis index scale, NRS scale, and WHOQOL-BREF were observed before treatment, after 2 weeks, and 4 weeks after treatment.

**Results:**

This study found that the osteoarthritis index scale and NRS scale of the shock wave group and the electroacupuncture group were lower than those before treatment; it had significant difference (*P* < 0.001). In WHOQOL-BREF, the shock wave group and the electroacupuncture group improved significantly four weeks after treatment (*P* < 0.001), which was statistically different from the conventional group (*P* = 0.04).

**Conclusion:**

Physical and rehabilitation medicine treatment (shock wave therapy) and traditional medical treatment (electroacupuncture) have better clinical effects on knee osteoarthritis, compared with conventional treatment. Shock wave and electric acupuncture have no apparent adverse reaction, suggesting that the treatment is safe and effective.

## 1. Background and Aim

Knee osteoarthritis (KOA) is a common chronic disease of osteoarthritis, with a relatively high incidence in the elderly. KOA can cause severe systemic physical symptoms such as joint pain, swelling, stiffness, and restricted mobility [1]. The number of patients with KOA worldwide is currently estimated to be as high as 350 million [2]. The prevalence of knee osteoarthritis is 8.1% in China [3]. KOA has become a serious public health problem that seriously affects the life and health of middle-aged and elderly people. Therefore, effective treatment of KOA has become a hot and difficult issue. Traditional Chinese acupuncture has a long history in the treatment of knee osteoarthritis. It has significant effects in relieving patients' pain and improving clinical symptoms, and even in repairing degenerative knee joints with simple, convenient, and easy operation [4–6]. Electroacupuncture (EA) is a form of acupuncture therapy that combines traditional acupuncture with electrical stimulation, which is famous for quantification and repeatability. Previous studies have confirmed the good therapeutic effect of electroacupuncture on KOA. The specific mechanisms include anti-inflammatory, improving blood circulation, and analgesia [7, 8]. In clinical biological research, Gang et al. [9]. found that electroacupuncture can improve the muscle tone of the rectus femoris in KOA patients, and Han and Sun [10] found that electroacupuncture can also improve the gait function of KOA patients. Traditional Chinese medicine can restore the mechanical balance of the knee joint to achieve a therapeutic effect by treating tendons or treating both muscles and bones at the same time. In addition to the direct improvement of muscle function, electroacupuncture also has a complex central analgesic mechanism. At the same time, electroacupuncture not only plays a direct role in improving muscle function but also has a complex central analgesic mechanism [11], which may play a direct anti-inflammatory effect on articular cartilage, resulting to treating pain and alleviating the degradation of KOA cartilage finally [12]. It has been proved that electroacupuncture can improve the atrophy of the rectus femoris and biceps femoris in KOA rabbit models. In addition, electroacupuncture had a protective effect on the articular cartilage of the rabbit KOA model. In recent years, some new methods of noninvasive treatment, such as extracorporeal shock wave, have emerged. Some studies have shown that the mechanism of pain improvement is that shock wave can incapacitate sensory unmyelinated fibers and reduce the expression of nociceptors on neurocutaneous calcitonin gene-related multiskin, thus reducing the pain sensitivity of patients [13]. When the shock wave acts on the local area, it causes minor trauma to the affected area, thus improving the blood supply to the local microcirculation. The levels of interleukin-1, tumor necrosis factor a, and nitric oxide in cartilage were decreased, while the subchondral bone mineral density was increased after extracorporeal shock wave intervention, which were proved that extracorporeal shock wave was beneficial in reducing cartilage inflammation and enhancing subchondral bone strength. The purpose of this study was to analyze the clinical efficacy, adverse reactions, and safety of rehabilitation therapy (shock wave therapy) and alternative medicine (traditional Chinese acupuncture electroacupuncture) in the treatment of knee osteoarthritis. This study provided a new idea of integrated rehabilitation medicine for the clinical treatment of knee osteoarthritis.

RETRACTED

## 2. Method

### 2.1. Subjects

This study retrospectively selected patients with knee osteoarthritis in the outpatient clinic from January 1, 2018, to December 30, 2020, and followed the necessary inclusion and exclusion criteria. Each participant signed an informed consent form before participation. This study approved by the Ethics Committee of the Central Hospital of Longhua District was conducted by the Central Hospital of Longhua District, Shenzhen.

Diagnostic criteria: defined the criteria for the diagnosis of knee osteoarthritis in 1995 by the American College of Rheumatology [14].

Inclusion criteria: (a) according to the Chinese “Guidelines for the Diagnosis and Treatment of Osteoarthritis,” the research subjects who can be clearly diagnosed as knee osteoarthritis; (b) the patients are all over 18 years old; (c) no other treatments have been used for the treatment of osteoarthritis in the past month; (d) informed consent was signed by the recruited patient.

Exclusion criteria: (a) patients with other serious bone and joint diseases, or diseases with similar clinical symptoms; (b) patients who have not signed the informed consent.

The included knee osteoarthritis patients were divided into the shock wave group (*n* = 54), electroacupuncture group (*n* = 41), and control group (*n* = 33) based on different treatments. In this study, the percentage of females is 47.1% and males 52.9% in the control group (mean age 55.84 ± 5.62 years; mean course of disease 4.35 ± 1.23 years); the percentage of females is 51.2% and males 48.8% in the electroacupuncture group (mean age 56.32 ± 5.78 years; mean course of disease 4.82 ± 1.57 years); the percentage of females is 48.1% and males 51.9% in the shock wave group (mean age 55.31 ± 5.54 years; mean course of disease 4.59 ± 1.49 years). The difference in basic population specificity was not statistically significant among the three groups. Please see Table 1.

### 2.2. Intervention

Each patient with knee osteoarthritis was treated for four weeks.

1. Shockwave group: shockwave treatment was performed on the basis of Voltaren topical treatment, once every 7 days, the frequency was 7 Hz, and there are 2000 hits each time. Extracorporeal shock wave therapy instrument (Brand: Swiss EMS, Model: Swiss DolorClast Classic)
2. Electroacupuncture group: electroacupuncture was performed on the basis of Voltaren topical therapy. Specific treatment method: use disposable 40 mm∗0.3 mm sterile acupuncture needles (Universal brand), select the affected side (Liangqiu ST34, Xuehai SP10), (Heding EX-LE2, Zusanli ST36), (EX-LE4) External calf nose ST35), (Yinlingquan SP9, Yanglingquan GB34) 4 sets of electroacupuncture, frequency 1 Hz, time 20 minutes, continuous wave, the size is subject to personal tolerance, and treatment is performed every other day (electroacupuncture instrument, Brand: Shantou Dajia, Model: 6805-AII)
3. Control group: Voltaren topical treatment. Manufacturer: Beijing Novartis Pharmaceutical Co., Ltd. Appropriate amount for external use, three times a day

Primary endpoints: The Western Ontario and McMaster Universities Osteoarthritis Index, WOMAC.

RETRACTED

Secondary endpoints: NRS and WHOQOL-BREF.

### 2.3. Evaluation

Western Ontario and McMaster Universities Osteoarthritis Index (WOMAC). (1) The Osteoarthritis Index Score Scale includes three dimensions: pain, stiffness, and difficulty in daily activities, and 24 survey items with a score of 0-96. The pain dimension in the scale contains 5 research survey items, the stiffness dimension in the scale contains 2 research survey items, and the difficulty of daily activities contains 17 research survey items. Each survey item has a score of 0-4. The higher the score, the more severe the disease, showing a positive correlation trend. (2) The Numerical Rating Scale (NRS) is used to evaluate the degree of pain in patients with knee osteoarthritis, and the score ranges from 0 to 10 points. In this clinical study, the patients themselves scored according to the degree of pain. The higher the score, the more severe the knee osteoarthritis pain. See Table 2 for details.

(3) Use the World Health Organization's Quality of Life Scale (WHOQOL-BREF) for scoring. Perform clinical evaluation based on changes in points. There are 26 questions in the scale, including 4 fields, namely, the physiological field, the psychological field, the social field, and the environmental field. The scale can generate scores in 4 fields, and field scores are recorded in a positive direction. The higher the score, the better the quality of life. The field score is obtained by calculating the average score of the item it belongs to and multiplying by 4. Physiological domain (PHYS) = 4 × [(6 − Q3) + (6 − Q4) + Q10 + Q15 + Q16 + Q17 + Q18]/7. Psychological domain (PSYCH) = 4 × [Q5 + Q6 + Q7 + Q11 + Q19 + (6 − Q26)]/6. Social domain (SOCIL) = 4 × (Q20 + Q21 + Q22)/3, and environmental domain (ENVIR) = 4 × (Q8 + Q9 + Q12 + Q13 + Q14 + Q23 + Q24 + Q25)/8.

RETRACTED

### 2.4. Statistical Analysis

Statistical analysis was performed using SPSS software 22.0. Quantitative data such as age (years), course of disease (years), osteoarthritis index score, and NRS were all described by statistics. Age, course of disease, osteoarthritis index score NRS, and WHOQOL-BREF score were statistically analyzed by one-way ANOVA LSD (satisfying the effect of homogeneity of variance) and T3 test (not satisfying the effect of homogeneity of variance). Differences were tested using pairwise *q*-tests. Repeated measurement analysis of variance is used to evaluate the trend of osteoarthritis index score and NRS score with the time of TCM treatment. *P* < 0.05 was considered as statistically significant.

## 3. Results

### 3.1. Osteoarthritis Index Score Analysis before and after Treatment

The knee osteoarthritis patients in the control group, the electroacupuncture group, and the shock wave group were scored on the osteoarthritis index before treatment, after 2 weeks of treatment, and after 4 weeks of treatment. There were no statistically significant differences in the total scores of pain and stiffness, daily activities, and osteoarthritis index scores before treatment. After 2 weeks of treatment and 4 weeks of treatment, the total scores of pain, stiffness, daily activities, and osteoarthritis index scores of knee osteoarthritis patients in the electroacupuncture group and shock wave group decreased compared with the control group, and they were statistically significant (*P* value < 0.05).

Repeated measures of variance were used to analyze the trend of changes in the osteoarthritis index scores of each group before treatment, 2 weeks after treatment, and 4 weeks after treatment. The results showed that the score showed a gradual downward trend over time, and it was statistically significant (*P* < 0.05). There was no statistically significant difference between the electroacupuncture group and the shock wave group. See Table 3 for details.

### 3.2. Analysis of NRS Scores before and after Treatment

The knee osteoarthritis patients in the control group, electroacupuncture group, and shock wave group were evaluated for NRS before treatment, 2 weeks after treatment, and 4 weeks after treatment. The results showed that there was no statistically significant difference in NRS scores between the three groups before treatment (*P* = 0.965). After 2 weeks and 4 weeks of treatment, the scores of patients with knee osteoarthritis in the electroacupuncture group and shock wave group were lower than those in the control group, and they were statistically significant (*P* < 0.001).

Repeated measures of variance were used to analyze the decline in NRS scores of each group before treatment, 2 weeks after treatment, and 4 weeks after treatment. The change of the decline over time was statistically significant (*P* < 0.001). The decline of NRS scores in the electroacupuncture group and shock wave group was greater than that of the control group. There was no statistically significant difference between the electroacupuncture group and the shock wave group. See Table 4 for details.

RETRACTED

### 3.3. Analysis of WHOQOL-BREF Scale after Treatment

The knee osteoarthritis patients in the control group, the electroacupuncture group, and the shock wave group were scored by WHOQOL-BREF before treatment and 4 weeks after treatment. The results showed that there was no statistically significant difference in the scores of the three groups before treatment. After 4 weeks of treatment, the physical, psychological, and social environment of each group changed significantly. The physiological and psychological scores of patients with knee osteoarthritis in the electroacupuncture group and shock wave group increased compared with those in the conventional group (*P* < 0.001). There was no statistical difference between the three groups after treatment. See Table 5 for details.

### 3.4. Adverse Reactions

There were no adverse reactions in the electroacupuncture group and shock wave group during the one-month treatment course. The treatment is safe and effective.

## 4. Discussion

This study found that electroacupuncture combined with drugs and shock wave combined with drugs are more effective than conventional drug treatment in terms of arthritis index. The curative effect increases with the prolonged treatment time. There was no statistical difference between electroacupuncture and shock wave drugs. Clinical studies have shown that this effect may be related to the downregulation of the expression of IL-1*β* and MMP-3 in the synovial fluid of KOA patients and the upregulation of the expression of SOD [15].

In terms of pain index, electroacupuncture combined with drugs and shock waves combined with drugs are more effective than conventional drug treatments. As the treatment time is extended, the efficacy increases. There was no statistical difference between electroacupuncture and shock wave drugs. Animal experiments have shown that this effect can adjust the metabolic environment of chondrocytes by reducing the content of IL-1*β* and TNF-*α* in articular cartilage, inhibit the catabolism of cartilage matrix, and inhibit cartilage degeneration, thereby reducing the damage of articular cartilage.

In addition, in terms of quality of life assessment, electroacupuncture combined with drugs and shock waves combined with drugs are more effective than conventional drug treatment in terms of physiological and psychological indexes. There was no statistical difference between electroacupuncture and shock wave drugs. There was no statistical difference with the conventional group in terms of social environment. There was no statistical difference between the groups before and after treatment. Studies have shown that electroacupuncture can effectively alleviate the symptoms of KOA. The mechanism of action may be related to downregulating the expression of AQP3 to regulate water transport, reduce the degradation of cartilage extracellular matrix, and reduce the destruction of articular cartilage.

RETRACTED

The mechanism of this experiment needs to be further studied and proved in the future.

## Figures and Tables

**Table 1:** Baseline data for the three general population groups.

Indicators	Control group (*n* = 33)	Electroacupuncture group (*n* = 41)	Shock wave group (*n* = 54)
Age (year)	55.84 (5.62)	56.32 (5.78)	55.31 (5.54)
Sex *n* (%)			
m	17 (52.9)	20 (48.8)	28 (51.9)
f	16 (47.1)	21 (51.2)	26 (48.1)
Course of disease (year)	4.35 (1.23)	4.82 (1.57)	4.59 (1.49)

**Table 2:** NRS scoring criteria.

NRS scoring criteria					
Pain scale	Score				
	0	1-3	4-6	7-9	10
	Painless	Mild pain	Moderate pain	Severe pain	Worst pain

**Table 3:** Score analysis of osteoarthritis index scores before treatment, after 2 weeks of treatment, and 4 weeks of treatment of the three groups (mean(SD)).

Index	Time	Control group (*n* = 33)	Electroacupuncture group (*n* = 41)	Shock wave group (*n* = 54)
Pain	Before treatment	12. (2.89)	12.20 (2.03)	12.23 (2.03)
	After 2 weeks of treatment	8.41 (2.31)	6.34 (2.43)	6.28 (2.52)
	After 4 weeks of treatment	6.29 (1.21)	4.33 (1.92)	4.11 (1.58)
	*P*	<0.001	<0.001	<0.001
Stiff	Before treatment	4.27 (1.01)	4.52 (1.38)	4.41 (1.26)
	After 2 weeks of treatment	3.41 (1.13)	2.02 (0.93)	2.10 (1.04)
	After 4 weeks of treatment	2.20 (1.29)	1.31 (1.21)	1.23 (1.25)
	*P*	<0.001	<0.001	<0.001
Daily activity	Before treatment	58.36 (4.81)	59.19 (3.12)	58.77 (3.95)
	After 2 weeks of treatment	43.21 (4.92)	39.18 (3.83)	38.22 (3.83)
	After 4 weeks of treatment	26.23 (3.19)	23.16 (4.28)	22.85 (3.31)
	*P*	<0.001	<0.001	<0.001
Total score	Before treatment	74.88 (5.27)	75.93 (5.31)	76.07 (5.14)
	After 2 weeks of treatment	55.03 (5.82)	47.57 (4.92)	46.44 (5.37)
	After 4 weeks of treatment	34.72 (3.29)	28.85 (2.96)	27.68 (3.04)
	*P*	<0.001	<0.001	<0.001

**Table 4:** NRS score analysis of the three groups before treatment, 2 weeks after treatment, and 4 weeks after treatment (mean(SD)).

Index	Time	Control group (*n* = 33)	Electroacupuncture group (*n* = 41)	Shock wave group (*n* = 54)
NRS score	Before treatment	6.23 (1.27)	6.24 (1.03)	6.25 (1.18)
	After 2 weeks of treatment	5.21 (1.02)	4.07 (1.23)	4.06 (1.19)
	After 4 weeks of treatment	4.07 (1.21)	3.19 (1.24)	3.22 (1.20)
	*P*	<0.001	<0.001	<0.001

RETRACTED

**Table 5:** NRS score analysis of the three groups before treatment, 2 weeks after treatment, and 4 weeks after treatment (mean(SD)).

Index	Time	Control group (*n* = 33)	Electroacupuncture group (*n* = 41)	Shock wave group (*n* = 54)
Physiology	Before treatment	10.45 (1.12)	10.20 (0.97)	10.33 (1.03)
	After 4 weeks of treatment	12.31 (1.28)	12.89 (1.33)	12.98 (1.40)
	*P*	<0.001	<0.001	<0.001
Psychology	Before treatment	10.06 (0.68)	10.33 (0.85)	10.39 (0.97)
	After 4 weeks of treatment	12.18 (1.23)	13.07 (1.10)	13.22 (1.26)
	*P*	<0.001	<0.001	<0.001
Society	Before treatment	13.19 (1.14)	12.89 (1.15)	13.06 (1.16)
	After 4 weeks of treatment	14.33 (1.15)	13.82 (1.31)	14.00 (1.26)
	*P*	<0.001	<0.001	<0.001
Environment	Before treatment	11.27 (0.94)	11.48 (1.05)	11.37 (1.01)
	After 4 weeks of treatment	12.52 (1.02)	12.64 (0.89)	12.77 (0.99)
	*P*	<0.001	<0.001	<0.001

## Data Availability

The data used to support the findings of this study are available from the corresponding author upon request.
